# A Protein from *Dioscorea polystachya* (Chinese Yam) Improves Hydrocortisone-Induced Testicular Dysfunction by Alleviating Leydig Cell Injury via Upregulation of the Nrf2 Pathway

**DOI:** 10.1155/2021/3575016

**Published:** 2021-11-30

**Authors:** Shiting Yu, Bing Han, Xin Xing, Yixuan Li, Daqing Zhao, Meichen Liu, Siming Wang

**Affiliations:** Jilin Ginseng Academy, Changchun University of Chinese Medicine, 1035 Boshuo Road, Changchun, Jilin Province, China

## Abstract

Leydig cell injury has been described as a primary driver of testicular dysfunction and is affected by oxidative stress. *Dioscorea polystachya* (Chinese yam) is used to improve testicular dysfunction in clinical and pharmacological research via its antioxidative activity, but the mechanisms underlying the beneficial effect of Chinese yam on testicular dysfunction and its suppression of Leydig cell oxidative damage remain unclear. In this study, we obtained a Chinese yam protein (DP1) and explored its effectiveness and possible mechanism in improving testicular dysfunction in vivo and in vitro. We established a testicular dysfunction model in rats using hydrocortisone (HCT). DP1 increased body weight and organ index, improved the deterioration in testicular morphology (including increasing the diameter of seminiferous tubules and thickness of germinal cell layers, inhibiting testicular cell apoptosis by increasing the Bcl-2/Bax ratio, and impeding collagen leakage by downregulating TGF-*β*1 and p-SMAD2/3 expression), and restored the testosterone content. In addition, DP1 enhanced the number of Leydig cells in rats and H_2_O_2_-induced TM3 Leydig cells, and the effect of DP1 on the apoptosis, fibrosis, and testosterone content of TM3 cells was similar to that observed in vivo. These changes were dependent on the regulation of oxidative stress, including significantly reduced intracellular 8-hydroxy-2-deoxyguanosine levels, enhanced superoxide dismutase activities, and decreased superoxide anion levels, which were confirmed via a superoxide overexpression system. Furthermore, we observed that DP1 promoted Nrf2 nuclear import and upregulated antioxidant factor expression in vivo and in vitro. However, Nrf2 silencing eliminated the ability of DP1 to increase the Bcl-2/Bax ratio, reduce the expression levels of TGF-*β*1 and p-SMAD2/3, and increase testosterone contents in H_2_O_2_-induced TM3 cells. In conclusion, DP1 reversed the HCT-induced testicular apoptosis and fibrosis and decreased testosterone contents by alleviating Leydig cell oxidative damage via upregulation of the Nrf2 pathway.

## 1. Introduction

Leydig cells, the primary site of androgen synthesis and secretion, are essential in establishing and maintaining the male testicular microenvironment [1, 2]. Leydig cell injury is a vital factor contributing to testicular dysfunction and is accompanied by diminished fertility and erectile ability [3, 4]. Glucocorticoids, such as hydrocortisone (HCT), are widely used for the treatment of multiple diseases because of their strong anti-inflammatory and immunosuppressive effects [5, 6]. However, long-term or excessive exposure to glucocorticoids may induce Leydig cell lose their normal morphology and function and eventually lead to testicular dysfunction, which is largely associated with the induction of apoptosis and fibrosis [7–9]. Therefore, inhibition of apoptosis and fibrosis would hinder Leydig cell injury, which can in turn effectively delay the initiation and progression of glucocorticoids-induced testicular dysfunction.

Although the precise pathogenesis of glucocorticoid-induced testicular dysfunction is still unclear, it is generally believed that oxidative stress plays a crucial role in this process. Oxidative stress is caused by generating excessive reactive oxygen species (ROS), which considers as an important factor in the induction of apoptosis [10–13]. Simultaneously, ROS overproduction induces organ fibrosis via activation of profibrosis signaling pathways, such as TGF-*β*1/SMAD pathway [14, 15]. More importantly, previous studies have shown that glucocorticoids induce ROS accumulation and reduce antioxidant enzyme activities, causing testicular redox imbalance [16, 17]. Therefore, protecting Leydig cells from oxidative stress is an undoubtedly effective approach for preventing and alleviating glucocorticoid-induced testicular dysfunction.

As a transcription factor that regulates the cellular oxidative stress response, nuclear factor erythroid 2-related factor 2 (Nrf2) plays a crucial role in the maintenance of intracellular redox homeostasis [18, 19]. Under oxidative stress, Nrf2 translocates to the nucleus and promotes the expression of antioxidant factors (such as heme oxygenase 1 (HO-1), NAD(P)H dehydrogenase [quinone] 1 (NQO1), and glutamate--cysteine ligase catalytic subunit (GCLC)) to protect cells against ROS [20, 21]. In addition, Nrf2 activation plays an essential role in regulating cell apoptosis and fibrosis. Previous studies confirmed that the resistance to oxidative stress and antiapoptotic effects of melatonin on H_2_O_2_-induced Leydig cells was largely diminished after the siRNA-mediated silencing of Nrf2 [22]. In diabetic nephropathy models, Nrf2 activation was required for bergenin to inhibit oxidative stress and TGF-*β*1 expression [23]. Thus, therapeutic approaches targeting the Nrf2 pathway to attenuate oxidative stress are undoubtedly beneficial for the prevention and treatment of Leydig cell injury.

*Dioscorea polystachya* (Chinese yam) is a traditional Chinese medicine that has been used to treat the male reproductive system for thousands of years in China [24, 25]. Recent pharmacological studies have shown that Chinese yam or its extract considerably improves testicular dysfunction, such as enhancing testosterone levels and increasing sperm numbers [26, 27]. Our previous study demonstrated that Chinese yam protein extract ameliorated testicular injury in HCT-induced erectile dysfunction rats and had a greater effect on oxidatively damaged TM3 cells than water decoction extract, water extraction, alcohol precipitation extract, and alcohol extract [9]. More importantly, the results of our study and previous reports all preliminarily confirmed that resistance to oxidative stress was involved in the protective effect of Chinese yam on testicular dysfunction. However, the main active ingredient in Chinese yam responsible for protecting against HCT-induced testicular dysfunction by inhibiting Leydig cell injury remains unclear, and the mechanism underlying the role of oxidative stress in this protection has not been elucidated.

Considering the key role of oxidative stress in glucocorticoid-induced testicular dysfunction, in the present study, we first obtained the Chinese yam protein DP1 and determined that its ameliorating effect on testicular dysfunction was associated with alleviating Leydig cell injury using a HCT-treated rat model and H_2_O_2_-induced TM3 cell model. Moreover, DP1 exhibited a strong attenuating effect on HCT-induced oxidative stress in rat testes, and the inhibition of Leydig cell injury by DP1 was dependent on a reduction in oxidative stress, which was demonstrated using a superoxide overexpression system in vitro. Mechanistically, DP1 activated Nrf2 to increase the Bcl-2/Bax ratio and inhibit the TGF-*β*1/SMAD2/3 pathway, which suppressed Leydig cell apoptosis and fibrosis and increased testosterone secretion to reverse HCT-induced testicular dysfunction.

## 2. Materials and Methods

### 2.1. Extraction, Isolation, and Purification of DP1

Chinese yam (*Dioscorea polystachya*) was purchased from Jiaozuo, Henan Province, and identified by Professor Zhe Wang of Changchun University of Chinese Medicine (taxonomic serial number: 810115). Chinese yam was homogenized with 20 mM Tris-HCl buffer (buffer A, pH = 7.4) at a 1 : 10 ratio and then extracted at 4°C for 2 h. The supernatant was mixed with ammonium sulfate until the saturation reached 65% and left at 4°C overnight. The obtained supernatant was lyophilized by freeze-drying (LABCONCO, KC, USA) and formulated into a 20 mg/ml solution using 20 mM Tris-HCl buffer (pH = 7.4). The sample was applied to a DEAE Sepharose FF column (XK 26/40, GE Healthcare, Marlborough, USA) connected to an Akta purifier (GE Healthcare, Marlborough, USA). The column was equilibrated with buffer A and stepwise eluted with buffer A and 20 mmol/L Tris-HCl+1 M NaCl (buffer B, pH = 7.4) using a linear gradient (0%–100% buffer B, 0–120 min) at a flow rate of 5 ml/min. Gel filtration of isolated proteins was performed on a Sephadex G25 column (XK 26/40, GE Healthcare, Marlborough, USA) with ultrapure water. The sample was obtained and lyophilized, producing DP1. The concentration and molecular mass of DP1 were detected using SDS-PAGE with Coomassie blue staining and the BCA assay (Beyotime, Shanghai, China), respectively.

### 2.2. Animals and Treatments

The experiment was approved by the Ethical Committee for Animal Research of Changchun University of Chinese Medicine (Certificate No. SYXK, Ji, 2018-0014). Six-week-old male Sprague Dawley rats (SPF, 180–200 g) were randomly divided into 2 groups: the control group (*n* = 10) and the model group (*n* = 20). After acclimation to the laboratory environment for one week, rats in the model group were gavaged with HCT (10 mg/kg, Runhong pharmaceutical, Henan, China) for 10 d and divided evenly into two groups. Ten rats were randomly selected from the model group and gavaged with DP1 (0.9 mg/kg) for 10 d, and the rest of the rats were fed a normal diet. After treatment, all rats were anesthetized with 3% pentobarbital sodium, and serum samples and testicular and epididymal tissues were collected.

### 2.3. Histological Study

Testicular tissues were cut into paraffin sections and stained with hematoxylin and eosin (HE, Beyotime, Shanghai, China) or a Masson kit (Sigma-Aldrich, MO, USA). Apoptotic cells in each group were measured using a TUNEL assay in accordance with the manufacturer's instructions (Roche Diagnostics, Indianapolis, USA). Immunohistochemical staining was performed with a 3*β*-HSD antibody. Images were acquired with a stereomicroscope (SMZ25, Nikon, Japan) and an EVOS FL Auto Cell Imaging System (Life Technologies, Carlsbad, USA) and analyzed with ImagePro (version 6.3).

### 2.4. Testosterone Content Determination

The testosterone level in serum samples was measured using enzyme-linked immunosorbent assay (ELISA) kits (Sinobestbio, Shanghai, China) in accordance with the instructions.

### 2.5. Cell Culture and Transfection

The Leydig cell line (TM3) was obtained from Procell Life Science & Technology Co., Ltd. (Wuhan, China). TM3 cells were cultured in TM3 cell culture medium (Procell, Wuhan, China) at 37°C. For RNA interference, TM3 cells were transfected with Nrf2 siRNA (100 nmol/L) or negative control siRNA for 48 h using ribo*FECT™* CP reagent (RIBOBIO, Guangzhou, China). The transfection efficiency was detected by real-time PCR.

### 2.6. Cell Viability Testing and Establishment of the Superoxide Overexpression System

TM3 cells were seeded in 96-well plates at a density of 2 × 10^4^ cells/ml and treated with 0.8 *μ*g/ml DP1 for 24 h, followed by H_2_O_2_ for 2 h to establish oxidative damage conditions. A CCK-8 assay was performed for cell viability. The absorbance at 450 nm was evaluated using a microplate reader. To establish the superoxide overexpression system, 0.005 U/mg xanthine oxidase (XO, Sigma-Aldrich, MO, USA) was added to each well for 8 h after H_2_O_2_ induction. The cell or culture supernatant was collected and used for subsequent experiments.

### 2.7. Apoptosis Assay

TM3 cells were seeded in 6-well plates at a density of 2 × 10^4^ cells/ml and treated as previously mentioned. Annexin V/FITC-PI double staining was performed to evaluate the degree of cell apoptosis in accordance with the manufacturer's instructions (Roche Diagnostics, Indianapolis, USA). Cell apoptosis was assayed by flow cytometry (Amnis, Millipore Sigma, USA).

### 2.8. Real-Time PCR

After treatment, the total RNA in TM3 cells was extracted using TRIzol Reagent (Sigma-Aldrich, MO, USA). cDNA was synthesized following the instructions of the TaKaRa DRR047A kit (Takara, Shiga, Japan), and then the expression levels of *Nrf2*, *HO-1*, *NQO1*, and *GCLC* were measured with a SYBR Green PCR Master Mix (Takara, Shiga, Japan) and iCycler-iQ Real-time PCR Detection System (Bio-Rad Laboratories, Hercules, USA). The specific primers were synthesized by Comate Bioscience Co., Ltd. (Changchun, China) and shown in Table 1.

### 2.9. Immunofluorescence Staining

After treatment, the cells in each well were fixed with 4% paraformaldehyde for 15 min, blocked with PBS containing 5% goat serum and 0.5% Triton-X-100 for 30 min, incubated with a TGF-*β*1 antibody (Bioworld, Shanghai, China; 1 : 200) overnight at 4°C, and then incubated with a secondary antibody at room temperature for 1 h. The nuclei were stained with DAPI in the dark for 5 min. Images were acquired with an EVOS FL Auto Cell Imaging System.

### 2.10. ELISA Study

After treatment, the cell culture supernatant in each group was collected and assayed for the testosterone level, 8-hydroxy-2-deoxyguanosine (8-OHdG) content, and superoxide dismutase (SOD) activity using ELISA kits in accordance with the instructions.

### 2.11. Dihydroethidium (DHE) Assay

After treatment, the cells in each well were washed twice with PBS, incubated with 5 *μ*mol/L DHE (Beyotime, Shanghai, China) in the dark for 30 min, and then washed with PBS to remove the excess dye. Images were acquired with an EVOS FL Auto Cell Imaging System.

### 2.12. Western Blotting

The testicular tissues and harvested cells were homogenized in RIPA buffer (Beyotime, Shanghai, China) supplemented with 1% PMSF (Beyotime, Shanghai, China), and protein concentrations were quantified using a BCA kit. Using lysis buffer, the samples were adjusted to contain equal amounts of protein. The proteins were separated by SDS-PAGE, transferred to nitrocellulose membranes, blocked with 5% skim milk, incubated with primary antibodies against Bcl-2, Bax, TGF-*β*1, p-SMAD2/3, Nrf2, and HO-1 (Bioworld, Shanghai, China) overnight at 4°C, and then incubated with HRP-conjugated secondary antibodies (Jackson Immuno Reseach, PA, USA) for 1 h. The blots were visualized with an ECL kit (Beyotime, Shanghai, China) and detected with an iBright™ FL1000 instrument (Thermo Fisher Scientific, Massachusetts, USA).

### 2.13. Statistical Analysis

The results were obtained by three independent experiments. All data were analyzed by one-way ANOVA, followed by the Tukey–Kramer multiple comparison test using GraphPad Prism software v6.0 and expressed as the mean ± S.D. *P* < 0.05 was considered statistically significant.

## 3. Results

### 3.1. Isolation, Purification, and Characteristics of DP1

In this experiment, DP1 was separated and purified by anion-exchange chromatography and gel filtration chromatography. DP1 presented as a single band in the SDS-PAGE gel shown in Figure 1(a), which suggested optimal separation of DP1. The molecular weight of DP1 was estimated to be approximately 13.2 kDa. The BCA method was used to detect and analyze the protein content of DP1. The standard curve equation of the line was *y* = 0.6727*x* + 0.0052 and *R*^2^ = 0.9991, and the protein concentration of DP1 was calculated to be 99.9%.

### 3.2. DP1 Ameliorated Testicular Dysfunction in HCT-Treated Rats

In vivo, HCT was used to stimulate the rats to mimic the testicular dysfunction observed in patients induced by high-dose glucocorticoid intake. We first observed that the rats induced with 10 mg/kg HCT exhibited a significant loss in body weight, testis index, and epididymis index (Table 1). After treatment with DP1, these values were substantially increased.

HE staining showed that the testes of HCT-treated rats exhibited morphological changes, including a large number of shrunken seminiferous tubules, vacuolization, and reduced thickness of germ cell layers (Figure 2(a) and Table 2). DP1 exhibited a significant ameliorating effect on these injuries. Apoptosis in testicular tissues was detected by the TUNEL assay. DP1 significantly decreased the expression of TUNEL in testicular cells of the HCT-treated rats (Figures 2(b) and 2(c)). The ratio of the Bcl-2/Bax protein expression is a critical indicator of apoptosis. Western blotting assays indicated that HCT decreased the Bcl-2/Bax ratio in testicular tissues, which was largely reversed by DP1 treatment (Figures 2(d) and 2(e)). In addition, DP1 significantly decreased the collagen leakage of testicular tissues in HCT-treated rats, which was detected by Masson staining (Figure 2(f)). We further investigated the expression of the TGF-*β*1/SMAD2/3 pathway, which regulates collagen production. The results revealed that DP1 almost completely blocked the HCT-enhanced expression of TGF-*β*1 and p-SMAD2/3 (Figures 2(e) and 2(g)).

To further verify whether HCT induces testicular function damage in rats, the testosterone content was measured. The results showed that the testosterone content in the HCT group was significantly decreased compared with the control group (Figure 2(h)). It is noteworthy that the inhibitory effect of HCT on testosterone almost disappeared after DP1 treatment.

### 3.3. Amelioration of Testicular Dysfunction by DP1 Was Related to the Restoration of Leydig Cells

Immunohistochemistry of testicular tissues with an antibody against 3*β*-HSD was performed to detect the amount of Leydig cells in rats (Figure 3(a)). Treatment with DP1 potently reversed the HCT-induced decline in Leydig cells. In vitro, H_2_O_2_ was used to stimulate the TM3 Leydig cell line to mimic the Leydig cell damage observed in patients induced by high-dose HCT intake. The CCK-8 assay results showed that DP1 evidently enhanced the viability of H_2_O_2_-induced TM3 cells (Figure 3(b)). The number of apoptotic TM3 cells detected by flow cytometry was obviously lower in the DP1 group than in the H_2_O_2_ group (Figures 3(c) and 3(d)). Moreover, DP1 increased the Bcl-2/Bax ratio in H_2_O_2_-induced TM3 cells (Figures 3(e) and 3(g)). Western bolt and immunofluorescence assays indicated that DP1 almost completely blocked the H_2_O_2_-enhanced protein expression of TGF-*β*1 and p-SMAD2/3 and decreased the fluorescence intensity of TGF-*β*1 in TM3 cells (Figures 3(f)–3(h)). In addition, the inhibition of testosterone contents by H_2_O_2_ was substantially reversed after DP1 treatment (Figure 3(i)).

### 3.4. Inhibition of Testicular Dysfunction by DP1 Was Dependent on the Reduction in Oxidative Stress in Leydig Cells

Oxidative stress is considered the main cause of excessive apoptosis and fibrosis in testicular cells, which subsequently leads to testicular dysfunction. As shown in Figures 4(a) and 4(b), stimulation with HCT obviously increased the 8-OHdG levels and decreased SOD activities in rats. DP1 significantly reversed these abnormal changes, similar to the effect observed in H_2_O_2_-induced TM3 cells. Immunofluorescence assay results indicated that the excessive increase in superoxide anion induced by H_2_O_2_ was markedly inhibited after DP1 treatment (Figure 4(c)). To investigate whether the beneficial effect of DP1 on Leydig cell injury was associated with reduced oxidative stress, a superoxide overexpression system was constructed using xanthine oxidase in TM3 cells. Importantly, treatment with xanthine oxidase not only further exacerbated the effects of H_2_O_2_ on TM3 cells, including inhibiting the expression of Bcl-2/Bax, elevating the expression of TGF-*β*1 and p-SMAD2/3, and reducing the testosterone content, but it also attenuated the beneficial effect of DP1 on H_2_O_2_-induced TM3 cells. Together, these findings imply that the DP1-mediated reduction in oxidative stress was involved in ameliorating Leydig cell injury (Figures 4(d)–4(f)).

### 3.5. DP1 Promoted the Upregulation of the Nrf2/HO-1 Pathway

As demonstrated by the Western blotting assays, DP1 intervention significantly promoted the expression levels of Nrf2 and its downstream protein HO-1 in the testes of testicular dysfunction rats (Figures 5(a) and 5(b)). In addition, real-time PCR assays revealed that DP1 exhibited a potent promoting effect on the mRNA levels of *HO-1*, *NQO1*, and *GCLC* in H_2_O_2_-induced TM3 cells (Figure 5(c)). Moreover, compared with the H_2_O_2_ group, DP1 evidently elevated the nuclear expression of Nrf2 and HO-1 but had no effect on the cytoplasmic expression of Nrf2 (Figures 5(d) and 5(e)).

### 3.6. Nrf2 Activation Was Required for DP1 to Inhibit Leydig Cell Injury

To further clarify the mechanism by which DP1 reduced oxidative stress and ameliorated testicular dysfunction, the influence of Nrf2 silencing on the effects of DP1 was determined in H_2_O_2_-induced TM3 cells. The transfection efficiency of the Nrf2 siRNA was confirmed (Figure 6(a)). We found that the ability of DP1 to increase Nrf2 and HO-1 protein expression and inhibit superoxide anion was significantly reduced after Nrf2 silencing (Figures 6(b)–6(d)). Moreover, the Nrf2 siRNA interfered with the inhibitory effect of DP1 on apoptosis and fibrosis by reducing the ratio of Bcl-2/Bax, enhancing the expression levels of TGF-*β*1 and p-SMAD2/3 and increasing the fluorescence intensity of TGF-*β*1 (Figures 6(e)–6(g)). In addition, the DP1-mediated increase in the testosterone content in H_2_O_2_-induced TM3 cells was largely diminished by Nrf2 siRNA transfection (Figure 6(h)).

## 4. Discussion

A previous study revealed that Chinese yam protein extract enhanced testosterone levels and attenuated testicular fibrosis and oxidative stress in HCT-induced erectile dysfunction rats and H_2_O_2_-treated TM3 cells, suggesting that Chinese yam protein is potentially effective for the treatment of testicular dysfunction via the inhibition of oxidative stress [9]. In the present study, we first extracted a protein (DP1) from Chinese yam and demonstrated that it effectively ameliorated HCT-induced testicular dysfunction by alleviating Leydig cell injury, including increasing cell numbers, inhibiting excessive apoptosis and fibrosis, and increasing the testosterone content. In addition, the molecular evidence indicated that HCT or H_2_O_2_ induced oxidative stress by elevating 8-OHdG levels and decreasing SOD activities and superoxide anion expression in vivo or in vitro, and these effects were attenuated by DP1 treatment. Furthermore, Nrf2 activation was involved in the protective effect of DP1 on Leydig cell injury. Thus, these results suggested that DP1 exhibited an ameliorating effect on HCT-induced testicular dysfunction by alleviating Leydig cell injury via activation of the Nrf2 pathway (Figure 7).

Researchers have found that testicular dysfunction induced by excessive HCT is characterized by disrupted testicular morphology and suppressed ability of the testes to produce testosterone [28, 29]. Regarding testicular morphology, the present study first demonstrated that DP1 effectively alleviated the HCT-induced decreases in testicular and epididymal index, seminiferous tubule atrophy, and reduced germ cell layer thickness in testicular tissue. In addition, excessive apoptosis and fibrosis contribute to abnormal testicular pathological morphology induced by glucocorticoids [9, 30]. Under the induction of HCT, the TUNEL expression in testicular tissues was significantly increased, and DP1 reversed the excessive apoptosis. Increasing the Bcl-2/Bax ratio is critical to block cell apoptosis [31, 32]. The current study demonstrated that Bcl-2/Bax was involved in the antiapoptotic effect of DP1 in the testes of the HCT group. In the testicular tissue, fibrosis can induce excessive deposition of collagen, which causes testicular lesions [33]. Our study proved that DP1 intervention attenuated the enhanced deposition of collagen fibers in the testicular interstitium of HCT-treated rats, which suggested that DP1 improved the testicular fibrosis induced by HCT. TGF-*β*1 plays a role in signal transduction during tissue recovery and fibrosis [14, 15, 34]. Specifically, it activates SMAD2/3 to form a complex by initiating intracellular signal cascades and regulates the excessive proliferation of collagen, which leads to tissue fibrosis [35]. The TGF-*β*1/Smad2/3 signaling pathway is a key regulatory mechanism that promotes the occurrence and development of testicular fibrosis [36]. We further explored the mechanism by which DP1 inhibited HCT-induced fibrosis in testicular cells and found that its positive regulatory effect was accomplished by reducing the expression levels of TGF-*β*1 and p-SMAD2/3. As one of the primary functions of the testes, testosterone secretion promotes spermatogenesis and male reproductive organ maturation and maintains secondary sexual characteristics and functions [37, 38]. In our study, we found that DP1 reversed the impaired testosterone secretion in rats induced by HCT. These results suggest that DP1 potentially alleviates HCT-induced testicular dysfunction by restoring testicular morphology and testosterone contents.

As one of the main functional cells that form the physiological structure of the testis, Leydig cells are primarily responsible for the synthesis and production of testosterone [39, 40]. Glucocorticoid-mediated testicular dysfunction is closely related to the destruction of Leydig cells, which is thought to be induced by the loss of cell numbers and excessive apoptosis [41, 42]. To test whether the effects of DP1 on testicular dysfunction were linked to restored Leydig cell numbers, the influence of DP1 on the number of Leydig cells was evaluated both in vivo and in vitro. Our study first found that DP1 reversed the HCT-induced decline in the number of Leydig cells in testicular tissues. Oxidative stress is a major factor contributing to glucocorticoid-induced toxic effects on organisms [43–45]. The testis is more susceptible to peroxidative damage due to its higher content of polyunsaturated fatty acids [46]. Moreover, our previous study has proved that Chinese yam has the similar protective mechanism between glucocorticoid-induced testicular dysfunction rats and H_2_O_2_-induced TM3 Leydig cell line [9]. Therefore, this study chose H_2_O_2_ to directly induce oxidative stress in the TM3 cells to mimic the damage caused by HCT in Leydig cells in vivo and further proved that DP1 relies on the resistance to oxidative stress against testicular dysfunction in vitro. Our results showed that DP1 promoted the viability of H_2_O_2_-treated TM3 cells, similar to the effects observed in vivo. Furthermore, consistent with its effects on the testicular tissues of HCT-treated rats, DP1 inhibited the apoptosis and fibrosis of TM3 cells induced by H_2_O_2_, through decreasing the number of apoptotic cells, enhancing the ratio of Bcl-2/Bax, and reducing the expression of TGF-*β*1 and TGF-*β*1/SMAD2/3. In addition, the testosterone contents in TM3 cells were obviously improved after treatment with DP1. These findings revealed that the amelioration of testicular dysfunction by DP1 was related to the restoration of Leydig cell number and function.

Although the pathological mechanism by which glucocorticoids induce testicular dysfunction is still unclear, testicular tissues are susceptible to oxidative stress, which might affect the normal physiological functions of the testis for the following reasons: (1) oxidative stress enhances the antioxidant status and inhibits lipid peroxidation in the testis [47]; (2) oxidative stress changes the normal histomorphology of the testes and elevates the germ cell apoptotic index by decreasing the expression of caspase-3 and the Bcl-2/Bax ratio [16, 30], and (3) oxidative stress affects organ fibrosis by regulating the TGF-*β*1/SMAD pathway and may be related to testicular fibrosis [9, 19, 48, 49]. In the current study, the increase in 8-OHdG levels and reduction in SOD activities in the testes of HCT-treated rats were consistent with the excess superoxide anion in H_2_O_2_-induced TM3 cells, both revealing that the testes were in a state of imbalance between free radicals and antioxidants. DP1 treatment relieved this imbalance and was an effective strategy for the attenuation of oxidative stress. Furthermore, a superoxide overexpression system in TM3 cells was established using xanthine oxidase to explore the relationship between DP1-alleviated Leydig cell injury and resistance to oxidative stress. The results showed that the attenuation effects of DP1 on Leydig cell apoptosis, fibrosis, and testosterone levels were significantly inhibited, implying that the beneficial effects of DP1 on the damaged Leydig cells were associated with reduced oxidative stress.

Nrf2, a central regulator of redox homeostasis, translocates to the nucleus under oxidative stress to activate the expression of antioxidant factors, such as HO-1, NQO1, and GCLC [50]. More importantly, activation of the Nrf2 signaling pathway is conducive to the restoration of testicular function [51–53]. This study found that DP1 enhanced the total protein expression of Nrf2 and HO-1 in testicular tissues of HCT-treated rats. In addition, DP1 promoted the nuclear translocation of Nrf2 in damaged TM3 cells, increased the protein expression of HO-1, and enhanced the transcription of HO-1, NQO1, and GCLC, thereby reducing the accumulation of superoxide anion. These results suggest that the Nrf2 pathway might be involved in the ability of DP1 to protect against HCT-induced testicular oxidative stress. Several studies have revealed that oxidative stress regulated by Nrf2 is closely related to cell apoptosis, fibrosis, and testosterone production. Knockdown of Nrf2 significantly potentiated TP-induced TM4 Sertoli cell apoptosis [54]. In addition, in diabetic nephropathy mice, Nrf2 activation was indispensable for the bergenin-mediated inhibition of oxidative stress and extracellular matrix generation [23]. Furthermore, in aging mice, Nrf2 knockout further reduced testosterone production [55]. Our results showed that Nrf2 silencing abrogated the effects of DP1 on H_2_O_2_-induced TM3 cells, including the enhancement of HO-1 expression and the reduction of superoxide anion levels. Moreover, siRNA knockdown of Nrf2 almost completely reversed the attenuation of DP1 on apoptosis and fibrosis effects, mainly through its influence on the Bcl-2/Bax ratio and TGF-*β*1/SMAD2/3 signaling pathway. The promoting effect of DP1 on the testosterone content was also impaired by Nrf2 silencing. The above results indicated that Nrf2 activation was required for DP1 to inhibit oxidative stress and testicular dysfunction. However, the importance of DP1 on the regulation of Nrf2 pathway in an in vivo testicular injury model still needs to be answered using a Nrf2 knockout model.

## 5. Conclusion

As far as we know, this is the first to prove that DP1 has a protective effect on HCT-induced testicular dysfunction. These findings revealed that DP1 ameliorated testicular dysfunction due to Leydig cells injury through inhibiting apoptosis and fibrosis and enhancing testosterone content in vivo or in vitro and is dependent on suppressing oxidative stress *via* Nrf2 pathway.

## Figures and Tables

**Figure 1:** The molecular weight of DP1.

**Figure 2:** DP1 ameliorated testicular dysfunction in HCT-treated rats. (a) Histomorphological changes in testicular tissues. (b, c) Apoptosis levels of testicular cells were detected by the TUNEL assay. (d, e) The ratio of Bcl-2/Bax in testicular tissues was detected by Western blotting. (f) Masson staining for collagen fibers in testicular tissues. (e, g) The protein expression levels of TGF-*β*1 and p-SMAD2/3 in testicular tissues were detected by Western blotting. (h) Comparison of the testosterone content in rats. Each bar represents the mean ± SEM. The images were captured at a magnification of ×100 or ×200. ^##^*P* < 0.01 and ^###^*P* < 0.001 vs. the control group; ^∗∗^*P* < 0.01 and ^∗∗∗^*P* < 0.001 vs. the HCT group.

**Figure 3:** Amelioration of testicular dysfunction by DP1 was related to the restoration of Leydig cells. (a) Immunohistochemistry with an antibody against 3*β*-HSD was performed to measure the amount of Leydig cells in testicular tissues of rats. (b) Effect of DP1 on the cell viability of TM3 cells detected by CCK-8 assays. (c, d) Flow cytometry was conducted to analyze the number of apoptotic TM3 cells. (e, g) The ratio of Bcl-2/Bax in TM3 cells was detected by Western blotting. (f, g) The protein expression levels of TGF-*β*1 and p-SMAD2/3 in TM3 cells were detected by Western blotting. (h) Immunofluorescence assays were performed to detect the expression of TGF-*β*1 in TM3 cells. (i) Comparison of the testosterone levels in TM3 cells. Each bar represents the mean ± SEM. All images were captured at a magnification of ×100. ^#^*P* < 0.05, ^##^*P* < 0.01, and ^###^*P* < 0.001 vs. the control group; ^∗^*P* < 0.05, ^∗∗^*P* < 0.01, and ^∗∗∗^*P* < 0.001 vs. the H_2_O_2_ group.

**Figure 4:** Inhibition of testicular dysfunction by DP1 was dependent on the reduction in oxidative stress in Leydig cells. (a) 8-OHdG levels and (b) SOD activities in testicular tissues. (c) Immunofluorescence staining was performed to measure the superoxide anion levels in TM3 cells. (d, e) The ratio of Bcl-2/Bax and the protein expression levels of TGF-*β*1 and p-SMAD2/3 in TM3 cells were detected by Western blotting. (f) Comparison of the testosterone levels in TM3 cells. Each bar represents the mean ± SEM. The images were captured at a magnification of ×100. ^#^*P* < 0.05, ^##^*P* < 0.01, and ^###^*P* < 0.001 vs. the control group; ^∗^*P* < 0.05 and ^∗∗∗^*P* < 0.001 vs. the HCT group or H_2_O_2_ group; ^^^*P* < 0.05 and ^^^^^*P* < 0.001 vs. the DP1 group. XO: xanthine oxidase.

**Figure 5:** DP1 promoted the upregulation of the Nrf2/HO-1 pathway. (a, b) The protein expression levels of Nrf2 and HO-1 in testicular tissues were detected by Western blotting. (c) Relative mRNA expression of HO-1, NQO1, and GCLC normalized to GAPDH in TM3 cells. (d, e) The protein expression levels of total Nrf2, nuclear Nrf2, and nuclear HO-1 in TM3 cells were detected by Western blotting. Each bar represents the mean ± SEM. The images were captured at a magnification of ×100. ^#^*P* < 0.05 and ^###^*P* < 0.001 vs. the control group; ^∗^*P* < 0.05, ^∗∗^*P* < 0.01, and ^∗∗∗^*P* < 0.001 vs. the HCT group or H_2_O_2_ group.

**Figure 6:** Nrf2 activation was required for DP1 to inhibit the Leydig cell injury. (a) Real-time PCR analysis of Nrf2 mRNA levels in TM3 cells transfected with Nrf2 siRNA or NC siRNA for 48 h. (b) Immunofluorescence staining was performed to measure the superoxide anion levels in TM3 cells. (c, d) The protein expression levels of Nrf2 and HO-1 in testicular tissues were detected by Western blotting. (e, f) The ratio of Bcl-2/Bax and the protein expression levels of TGF-*β*1 and p-SMAD2/3 in TM3 cells were detected by Western blotting. (g) Immunofluorescence analysis of TGF-*β*1 expression in TM3 cells. (h) Comparison of the testosterone levels in TM3 cells. Each bar represents the mean ± SEM. All images were captured at a magnification of ×100. ^##^*P* < 0.01 and ^###^*P* < 0.001 vs. the control group; ^∗^*P* < 0.05, ^∗∗^*P* < 0.01, and ^∗∗∗^*P* < 0.001 vs. the DP1 group.

**Figure 7:** Working hypothesis for the mechanism by which DP1 improves testicular dysfunction by alleviating Leydig cells injury via upregulation of the Nrf2 pathway.

**Table 1:** Primer sequences for quantitative real-time PCR.

Gene	Genebank number	Primer sequence (5′-3′)	Product size (bp)
*GAPDH*	NM_001289726.1	F: TGTTTCCTCGTCCCGTAG	108
		R: CAATCTCCACTTTGCCACT	
*Nrf2*	NM_010902.4	F: AGCAGGACATGGAGCAAGTT	176
		R: TTCTTTTTCCAGCGAGGAGA	
*HO-1*	NM_010442.2	F: CCCACCAAGTTCAAACAGCTC	101
		R: AGGAAGGCGGTCTTAGCCTC	
*NQO1*	XM_036153810.1	F: AGCCCAGATATTGTGGCCG	101
		R: CCTTTCAGAATGGCTGGCAC	
*GCLC*	NM_010295.2	F: ACATCTACCACGCAGTCAAGGACC	134
		R: CTCAAGAACATCGCCTCCATTCAG	

**Table 2:** DP1 improved body weight, organ index, and parameters of testicular health in HCT-treated rats.

	Control	HCT	DP1
Body weight (g)	347.21 ± 7.43	298.61 ± 19.50^###^	337.98 ± 13.61^∗∗∗^
Testicular index (mg/g)	10.08 ± 0.54	8.30 ± 0.79^###^	9.25 ± 0.67^∗^
Epididymal index (mg/g)	3.26 ± 0.20	2.82 ± 0.22^###^	3.10 ± 0.21^∗^
Diameter of seminiferous tubules (*μ*m)	308.85 ± 2.45	278.09 ± 7.21^##^	302.97 ± 4.25^∗^
Germinal cell layer thickness (*μ*m)	68.14 ± 2.52	39.98 ± 6.07^###^	64.66 ± 1.82^∗∗∗^

^##^ *P* < 0.01 and ^###^*P* < 0.001 vs. the control group; ^∗^*P* < 0.05 and ^∗∗∗^*P* < 0.001 vs. the HCT group.

## Data Availability

All data used to support the findings of this study are included within the article.
